The article "Utilizing Machine Learning Techniques to Predict the Efficacy of Aerobic Exercise Intervention on Young Hypertensive Patients Based on Cardiopulmonary Exercise Testing" was published in 2021. Journal: J Healthc Eng.

# Utilizing Machine Learning Techniques to Predict the Efficacy of Aerobic Exercise Intervention on Young Hypertensive Patients Based on Cardiopulmonary Exercise Testing

**DOI:** 10.1155/2021/6633832

**Published:** 2021-04-21

**Authors:** Fangwan Huang, Xiuyu Leng, Mohan Vamsi Kasukurthi, Yulong Huang, Dongqi Li, Shaobo Tan, Guiying Lu, Juhong Lu, Ryan G. Benton, Glen M. Borchert, Jingshan Huang

**Affiliations:** ^1^College of Mathematics and Computer Science, Fuzhou University, Fuzhou 350108, China; ^2^Department of Cardiology, First Affiliated Hospital of Sun Yat-sen University, Guangzhou 510080, China; ^3^School of Computing, University of South Alabama, Mobile, AL 36688, USA; ^4^College of Allied Health Professions, University of South Alabama, Mobile, AL 36688, USA; ^5^Department of Pharmacology, College of Medicine, University of South Alabama, Mobile, AL 36688, USA

## Abstract

Recently, the incidence of hypertension has significantly increased among young adults. While aerobic exercise intervention (AEI) has long been recognized as an effective treatment, individual differences in response to AEI can seriously influence clinicians' decisions. In particular, only a few studies have been conducted to predict the efficacy of AEI on lowering blood pressure (BP) in young hypertensive patients. As such, this paper aims to explore the implications of various cardiopulmonary metabolic indicators in the field by mining patients' cardiopulmonary exercise testing (CPET) data before making treatment plans. CPET data are collected “breath by breath” by using an oxygenation analyzer attached to a mask and then divided into four phases: resting, warm-up, exercise, and recovery. To mitigate the effects of redundant information and noise in the CPET data, a sparse representation classifier based on analytic dictionary learning was designed to accurately predict the individual responsiveness to AEI. Importantly, the experimental results showed that the model presented herein performed better than the baseline method based on BP change and traditional machine learning models. Furthermore, the data from the exercise phase were found to produce the best predictions compared with the data from other phases. This study paves the way towards the customization of personalized aerobic exercise programs for young hypertensive patients.

## 1. Introduction

As a prevalent chronic disease, hypertension has been widely considered as a major risk factor for cardio-cerebrovascular events [1]. Strikingly, hypertension incidence is increasing most dramatically in young adults [2, 3]. As an alternative to antihypertensive drugs, lifestyle adjustments, including body weight control, diet, and exercise, can also be used to lower blood pressure (BP) [4, 5]. In particular, aerobic exercise not only directly reduces BP but also indirectly achieves similar effects by controlling body weight, reducing stress, and improving vascular endothelial function, along with other mechanisms [6–8]. Therefore, aerobic exercise intervention (AEI) has been widely recommended for the treatment of hypertension [9, 10]. Unfortunately, specific guidelines for effectively administering aerobic exercise aimed at antihypertension have not been widely accepted as there is significant individual variation in BP lowering achieved by the same exercise program, with the same exercise type, time, frequency, and duration [11–13]. Understanding the individual responsiveness to AEI before formulating comprehensive hypertension management plans will help to improve both effectiveness and efficiency of BP management. To our knowledge, research in this field is still very limited, thus motivating us to perform the work conducted in this paper.

For the clinical feasibility and practicality, this work provided an investigation on the feasibility of utilizing machine learning techniques to predict the efficacy of AEI on young hypertensive patients. Taking into account the prognostic ability of key cardiopulmonary variables, data mining was performed based on the data generated by cardiopulmonary exercise testing (CPET) before treatment. CPET provides a comprehensive physiological assessment of multiorgan system function, including not only cardiovascular and pulmonary but also musculoskeletal and hematopoietic systems [14]. It can help clinicians identify the severity of the disease and evaluate the response to treatments, thus playing an important role in formulating aerobic exercise training prescription and cardiac rehabilitation [15, 16]. In this paper, CPET being used is an electric bicycle with many sensors (see Figure 1) as the main ergometer to measure the changes of various cardiopulmonary metabolic indicators over time. To provide the best measure of the response to exercise, these data were collected “breath by breath” by an oxygenation analyzer attached to a mask. The specific test scheme guided by clinicians included four phases: (1) resting for 1 minute to relieve the patient's tension; (2) load-free cycling (no resistance on the pedals) for 3 minutes to warm up; (3) exercise for 5–12 minutes with increasing resistance on the pedals (20–35 watt/min increment) until maximal exertion; and (4) recovery for 6 minutes with the first 3 minutes of load-free cycling and the second 3 minutes of sitting still.

Based on the professional advice of clinicians, this paper first utilized a simple method as the baseline to predict the BP-lowering effect of AEI for young hypertensive patients. Just to be clear, BP in this paper was equal to the sum of systolic blood pressure (SBP) and diastolic blood pressure (DBP). This method compared BP at the 6th minute of recovery (R6BP) with BP at the pre-exercise resting (PEBP) in a single CPET before AEI. Patients with R6BP ≤ PEBP were predicted to be strong responders to AEI. If the converse was true, they were predicted to be weak responders. Subsequent experiments showed that the accuracy of this method was typically 50%–60%, closely approximating a random guess, and far beneath the requirement for making effective and accurate clinical exercise prescriptions. To meet this challenge, machine learning techniques were utilized to fully capitalize on the information present within several cardiopulmonary metabolic indicators provided by CPET. As such, this work provides useful insights into the formulation of personalized AEI prescriptions for young hypertensive patients. The main contributions of this paper are as follows:

- A sparse representation classifier based on analytic dictionary learning was designed to accurately predict the efficacy of AEI on BP lowering. This model can not only alleviate the interference of redundant information and noise brought by breath-by-breath collection but also overcome the deficiency of the existing sparse representation-based classifier which needs a large number of training samples.
- The significance of various cardiopulmonary metabolic indicators at different phases of CPET for this task was discussed through comparative experiments. The results showed that the data from the exercise phase can produce the best predictions compared with the data from other phases. Among various metabolic indicators, oxygen pulse (i.e., oxygen intake per heartbeat) was recommended as a powerful indicator for predicting the individual responsiveness to AEI.

The remainder of the paper is structured as follows.  Section 2 introduces various metabolic indicators of CPET used in this paper.  Section 3 briefly introduces the related works, including the development of application scenarios and research methods.  Section 4 describes the designed model in detail based on the shortcomings of the existing model.  Section 5 reports the experimental results along with analyses. Finally, conclusions and future works are summarized in Section 6.

## 2. Main Metabolic Indicators of CPET

CPET provides time-varying information regarding multiple indicators related to circulation, respiration, and gas metabolism at different levels of exercise intensity [17]. The nine indicators recommended by professional clinicians for this work are briefly described in the following:

1. Heart rate (HR): the number of heartbeats per minute. Normally, HR is 60–100 beats per minute at rest. HR varies individually according to age, sex, and other physiological factors.
2. Stroke volume (SV): the volume of blood ejected from either ventricle of the heart in a single beat. The main affecting factors of SV are myocardial contractility, venous return blood volume (preload), arterial BP (afterload), and so forth.
3. Cardiac output (CO): the volume of blood that flows out of the heart in a given period, usually denoted as liters per minute. It can be obtained by multiplying the average SV per beat by HR, varying with metabolism and activity. For example, it increases with muscle movement, emotional agitation, pregnancy, and so forth.
4. Oxygen pulse (VO_2_/HR): the volume of the oxygen intake per heartbeat. Hence, it is the amount of oxygen that the tissues of the body extract from oxygen carried by each SV. A higher oxygen pulse suggests better cardiopulmonary function. This can be used as a comprehensive index to determine the cardiopulmonary function.
5. Oxygen consumption/kilogram (VO_2_/kg): the volume of oxygen consumed by the metabolic processes of the body over a period of time, usually denoted as milliliters of oxygen per kilogram of body weight per minute. It reflects the body's ability to use oxygen and is usually determined by the maximum cardiac output, arterial oxygen content, cardiac output to the distribution index of the exercise muscle, and muscle oxygen capacity.
6. Tidal volume (VT): the volume of air inhaled or exhaled during a normal breath. It is related to age, sex, volume and surface, breathing habits, body metabolism, and so forth.
7. Ventilation volume/minute (VE): the volume of air inhaled or exhaled from the lungs in a minute, which can be obtained by multiplying VT by the respiratory rate.
8. Respiratory exchange ratio (R): the ratio of the carbon dioxide (CO_2_) output to the oxygen (O_2_) uptake (i.e., VCO_2_/VO_2_) during the same period. It reflects not only the exchange of tissue metabolism of gas but also the influence of transient change in gas storage.
9. Carbon dioxide ventilation equivalent (VE/VCO_2_): the ability of the body to discharge carbon dioxide, calculated as the ratio between the required ventilation volume and carbon dioxide output.

To illustrate the characteristics of these indicators more vividly, Figure 2 shows a visualization of the above nine indicators for a patient during the exercise phase of a CPET before AEI. Since each breath represents a sampling point, the information of each metabolic indicator collected by the breath-by-breath technique can be stored as a time series [18].

## 3. Related Works

CPET is a dynamic, noninvasive diagnostic method to evaluate cardiopulmonary function during increasing load exercise. Recently, the application of CPET in clinical decision-making for various diseases has been significantly developed. For example, CPET is playing a growing role in cardiology, including heart failure, valve diseases, and ischemic heart disease [19]. Buys et al. evaluated the predictive value of CPET for the incidence of hypertension in patients undergoing aortic coarctation surgery and determined the high-risk boundary as VE/VCO_2_ slope ≥27 and peak SBP ≥220 mmHg through Cox regression analysis [20]. Keller et al. suggested that BP overresponse in CPET might be a diagnostic tool for identifying high-risk groups of hypertension [21]. Besides, CPET can be used as a tool for preoperative risk stratification of patients (not limited to cardiopulmonary surgery) to predict postoperative adverse outcomes [22, 23]. Currently, one of the most impressive advances is that the integration of CPET and other tests has been introduced to diagnose several diseases [24]. Exercise stress echocardiography and CPET have been successfully combined in the dynamic assessment of heart failure for hypertensive patients [25]. Similarly, CPET combined with echocardiography of the right ventricle was applied to predict the prognosis of patients with pulmonary arterial hypertension [26].

From the perspective of research methods, in addition to traditional statistical analysis, data mining of CPET using machine learning techniques is gradually becoming a research hotspot. Leopold et al. developed a greedy heuristic algorithm based on feature clustering to study the ability of CPET to predict the anaerobic mechanical power outputs [27]. Braccioni et al. used a random forest algorithm to analyze the relationship between symptoms and cardiopulmonary parameters of lung transplant recipients based on incremental CPET [28]. Sakr et al. evaluated the performance of six machine learning techniques in predicting the individuals at risk of hypertension through treadmill stress tests on a massive crowd [29]. Unfortunately, the above work only selected some special values of cardiopulmonary metabolic indicators (such as peaks or slope) as features for analysis, without taking into account their time-varying characteristics. Our previous work has proved that time-varying data of some metabolic indicators obtained through CPET could be used to predict the efficacy of AEI [30], but how to further improve the predictive accuracy is still a challenge, especially in the case of insufficient training samples. This encourages us to perform the research conducted in this paper.

In fact, the prediction of the BP-lowering effect of AEI by using a certain metabolic indicator can be transformed into time series classification (TSC) for data mining. To date, researchers have proposed hundreds of approaches for TSC in different application scenarios. TSC algorithms can be roughly divided into seven categories: (1) the whole-series-based method, (2) the interval-based method, (3) the shaped method, (4) the word-frequency-based method, (5) the model-based method, (6) the integration-based method, and (7) the deep learning-based method. Bagnall et al. evaluated the latest progress of TSC algorithms on 85 datasets in the University of California, Riverside (UCR) archive [31]. They recommended 1-nearest neighbor with dynamic time warping (1NN-DTW) and random forest (RF) as the baseline classifiers for comparison with other classifiers. Besides, they also concluded that the integration-based method can achieve high accuracy by utilizing multiple classifiers on one or more feature spaces. For example, Bagnall et al. integrated 35 classifiers on the time, frequency, change, and shapelet transformation domains [32]. On this basis, Lines et al. added two new classifiers, two additional transformation domains, and a hierarchical structure of probability voting to further improve the performance [33]. Recently, the method based on deep learning has gradually become a research hotspot [34]. Deep learning is characterized by learning hidden and more abstract representations of data from the original time series to achieve better classification performance. This method is widely used for end-to-end learning including methods such as convolutional neural networks (CNNs) [35] and echo state network (ESN) [36]. The common disadvantage of these methods is that they require a large amount of data and computational cost for model training. As this work represents the first stage in a larger experiment, the relatively small number of samples means that the above approach is not appropriate. Moreover, the robustness of the method to signal-to-noise ratio also needs to be considered because the process involved in collecting CPET data is usually very noisy. For the above reasons, a classifier based on sparse representation is recommended for the task in this paper.

## 4. Sparse Representation-Based Classifier

In this section, a sparse representation classifier based on dictionary learning was designed to accurately predict the efficacy of AEI on BP lowering. This method firstly eliminated redundant information and reduced noise by feature extraction based on the sparse representation. At the same time, it took advantage of learning of an analytic dictionary without requiring as many training samples as the existing sparse representation-based classifier.

### 4.1. Brief Introduction for Sparse Representation

Recently, sparse representation has received increasing attention in many fields. While initially developed for use in image analysis and signal processing, sparse representation has been successfully utilized for dealing with more general tasks in the machine learning field [37]. Specifically, given a signal *x* ∈ *R*^*m*^ of *m* observations and an overcomplete dictionary *D* ∈ *R*^*m*×*n*^ (*n* ≫ *m*) in which the column vector *d*_*i*_ (1 ≤ *i* ≤ *n*) is known as an atom, the main goal of the sparse representation is the reconstruction of a signal perfectly with the least possible number of atoms. Its objective function is as follows:

(1) $$\begin{array}{c} \min_{\alpha }{\left\|\alpha \right\|}_{0}\;s\mathrm{.t}\text{. }x=D\alpha \;, \end{array}$$

where *α* ∈ *R*^*n*^ is the sparse representation (or sparse solution) of *x* and ‖·‖_0_ refers to the number of nonzero elements in *α*. Due to the noise in the real signal, the solution of equation (1) can be approximated by either of the following two equations:

(2) $$\begin{array}{c} \min_{\alpha }{\left\|\alpha \right\|}_{0}\;s\mathrm{.t}.\;{\left\|x-D\alpha \right\|}_{2}^{2}\;\leq \delta , \end{array}$$

(3) $$\begin{array}{c} \min_{\alpha }{\left\|x-D\alpha \right\|}_{2}^{2}\;s\mathrm{.t}\text{. }{\left\|\alpha \right\|}_{0}\;\leq k, \end{array}$$

where *δ* can be considered as noise or a reconstruction residual; the sparse factor *k* is a predefined integer not less than 1. Besides, based on the Lagrange multiplier theorem, solving sparse representation can be equivalently transformed into an unconstrained minimization problem:

(4) $$\begin{array}{c} \min_{\alpha }{\left\|x-D\alpha \right\|}_{2}^{2}+\lambda {\left\|\alpha \right\|}_{0}, \end{array}$$

where *λ* is a positive constant used to achieve a tradeoff between the reconstruction residual and the sparse solution.

It should be noted that since obtaining the optimal solution with *l*_0_-norm minimization is an NP-hard problem, many algorithms have been proposed to deal with it. The strategies commonly used in these algorithms mainly include greedy pursuit strategy and convex relaxation strategy [38, 39]. The greedy pursuit strategy represented by the orthogonal matching pursuit (OMP) algorithm is to gradually approach the optimal solution through the sequential selection of column vectors (atoms) until the end of iteration [40]. For the convex relaxation strategy, the main idea is to replace the *l*_0_-norm minimization term with the *l*_1_-norm minimization term. Taking equation (3) as an example, it can be approximately equivalent to the lasso problem:

(5) $$\begin{array}{c} \min_{\alpha }{\left\|x-D\alpha \right\|}_{2}^{2}\;s\mathrm{.t}\text{. }{\left\|\alpha \right\|}_{1}\;\leq \varepsilon , \end{array}$$

where ‖·‖_1_ represents the sum of the absolute values of nonzero elements in *α* and *ε* is a positive constant given beforehand. The advantage of this strategy is that the *l*_1_-norm minimization problem has an analytical solution and can be effectively solved by several methods, such as least angle regression (LAR) [41], coordinate descent algorithm (CDA) [42], iterative shrinkage-thresholding algorithm (ISTA) [43], and many variations of them.

### 4.2. The Existing Sparse Representation-Based Classifier

Proposed by Wright et al., a sparse representation-based classifier (SRC) was first applied in the field of face recognition and then successfully extended to TSC [44, 45]. Specifically, the sparse representation of an unlabeled sample is first solved based on the dictionary composed of all labeled samples. Then, the reconstruction residuals of each class are calculated by using the samples of each class and the corresponding elements in the sparse representation. Finally, the classification is performed by examining which class leads to the minimum residual of the unlabeled sample. The steps to implement SRC are as follows:

(1) The *l*_2_-norm normalization is preprocessed for each sample of the whole dataset with a class number of *c.*
(2) A dictionary *D* = [*D*_1_, ⋯, *D*_*j*_, ⋯, *D*_*c*_] is generated, where *D*_*j*_ (1 ≤ *j* ≤ *c*) is a subdictionary composed of *j*th-class normalized samples in the training set as column vectors (atoms).
(3) The sparse representation *α* of the unlabeled sample *y* is obtained by using the algorithm described above.
(4) The unlabeled sample *y* is reconstructed, respectively, using each *D*_*j*_ and corresponding *α*_*j*_, where *α*_*j*_ (1 ≤ *j* ≤ *c*) is a subvector consisting of the elements in *α* corresponding to all atoms in *D*_*j*_. The label is determined based on the minimum residual, as shown in the following equation:
  (6) $$\begin{array}{c} \;{\text{Label}}_{y}={\text{class}}_{j}\;s\mathrm{.t}\text{. }\forall \;1\leq i\leq c\text{ and }i\neq j,\;\;{\left\|y-D_{i}\alpha_{i}\right\|}_{2}^{2}>{\left\|y-D_{j}\alpha_{j}\right\|}_{2}^{2}. \end{array}$$

Figure 3 shows the SRC schematic for a two-class problem. The success of the SRC depends on the hypothesis that the unlabeled sample can be best reconstructed by a linear representation of samples within the same class. However, once the samples of different classes look similar to each other, the performance of SRC is very unstable [46]. Besides, the dictionary cannot satisfy the overcompleteness if the number of labeled samples is less than the dimension of samples, which will also affect the performance of the SRC [47]. To overcome the shortcoming of the SRC, a sparse representation classifier based on an analytic dictionary was designed, and then its accuracy was improved by using dictionary learning. For the sake of simplicity, the model was called SRC-AL for short. The principle is described in the following.

### 4.3. The Designed Sparse Representation-Based Classifier

In the application domain of sparse representation, an overcomplete dictionary can be usually generated using data implementation or analytic approach [48]. The approach based on data implementation is to construct an explicit dictionary directly by using the raw data. This is exactly the way adopted by the SRC, intending to obtain the residuals of the unlabeled sample reconstructed by the samples of different classes. Unlike SRC, SRC-AL generates an implicit dictionary based on the analytic approach as the initial dictionary. This approach generally utilizes some fixed transformations, such as discrete Fourier transform (DFT), discrete cosine transform (DCT), and discrete wavelet transform (DWT) [49]. Compared to the data implementation, the analytic approach has the advantage of allowing an overcomplete dictionary of any size without being limited by the number of labeled samples. However, due to the poor adaptability, the analytic dictionary often requires further optimization through dictionary learning. K-singular value decomposition (K-SVD) is a popular algorithm for dictionary learning, which updates the used atoms one by one in an iterative manner to train the overcomplete dictionary most suitable for the training set [50].

Inspired by the sparse representation predictor for time series proposed by our previous work [51], the workflow of SRC-AL consists of the following six steps:

(1) Generate an initial dictionary *D* ∈ *R*^(*m*+*c*)×*n*^ by utilizing the analytic approach, where *m* is the dimension of the sample, *c* is the number of classes, and *n* is an arbitrary integer much larger than (*m* + *c*). The upper and lower parts of the dictionary are represented by *D*_*up*_∈*R*^*m*×*n*^ and *D*_*lw*_∈*R*^*c*×*n*^, respectively.
(2) Normalize each sample of the training dataset with *l*_2_-norm, and convert its label into one-hot encoding. Combine the above two parts into the new training sample *x*∈*R*^(*m*+*c*)^.
(3) According to the training set composed of new samples, update the initial dictionary through dictionary learning, with the purpose of better reconstructing the samples. The objective function of dictionary learning can be described as
  (7) $$\begin{array}{c} \underset{\alpha^{i},D}{\min}\;\overset{r}{\underset{i=1}{\sum }}{\left\|x^{i}-D\alpha^{i}\right\|}_{2}^{2}\\ \text{s.t }.\;{\left\|\alpha^{i}\right\|}_{0}\leq k, \end{array}$$
where *r* is the number of samples in the training set and *α*^*i*^ is a sparse representation of sample *x*^*i*^.
(4) Normalize the unlabeled sample *y*∈*R*^*m*^ with *l*_2_-norm, and then obtain its sparse representation *α*_*y*_ ∈ *R*^*n*^ based on the upper part of the learned dictionary (*D*_*up*_*'*  ∈ *R*^*m*×*n*^).
(5) Multiply the lower part of the learned dictionary (*D*_*lw*_'  ∈ *R*^*c*×*n*^) by the sparse representation *α*_*y*_ ∈ *R*^*n*^ to obtain the label vector *L*_*y*_∈*R*^*c*^.
(6) Determine the label of *y* according to the index of the element with the largest absolute value in *L*_*y*_, as shown in the following equation:
  (8) $$\begin{array}{c} {\text{Label}}_{y}={\text{class}}_{j}\;s\mathrm{.t}.\;\forall \;1\leq i\leq c\text{ and }i\neq j,\;\;\left|L_{y}\left(i\right)\right|<\left|L_{y}\left(j\right)\right|, \end{array}$$
where *L*_*y*_(*i*) represents the *i*th element in vector *L*_*y*_.

Figure 4 shows the SRC-AL schematic for a two-class problem. Assuming that sample *x*_1_ belongs to class 1, the green-filled blocks represent the normalized sample, and the following “10” represents the one-hot encoding of the label. Similarly, the blue-filled blocks represent the normalized sample of class 2, and the following “01” represents the one-hot encoding of its label. The dictionary filled with orange is generated by the analytic approach. To better reconstruct all training samples, a dictionary-learning algorithm (such as K-SVD) should be applied to constantly update the dictionary. Based on the upper part of the learned dictionary (*D*_*up*_'), the sparse representation *α*_*y*_ of the unlabeled sample *y* (grey-filled blocks) is solved, and then *D*_*lw*_'  × *α*_*y*_ is used to obtain the label vector *L*_*y*_. Finally, the element with the largest absolute value in *L*_*y*_ is set to 1, and the other elements are set to 0. This one-hot encoding is used to replace the question mark in Figure 4 to achieve the classification of *y*.

## 5. Experiments and Results

CPET data from 24 young patients with stage I hypertension before AEI treatment were used for the experiments. The dataset was provided by the Department of Cardiology, First Affiliated Hospital of Sun Yat-sen University, China. The whole exercise process of all the people was completed under the supervision of professional medical staff in the hospital. Blood pressure before and after exercise was assessed using both dynamic and exercise blood pressure results. Although the cost of each sample is very large, the data are highly comparable and reliable due to the guaranteed amount of exercise and more comprehensive monitoring indicators.

The performance of various machine learning models based on the data from the exercise phase was compared with the baseline method given by the clinician. Note that the baseline method only focused on BP change between pre-exercise and postexercise within a single CPET, while the machine learning model took into account the time series of metabolic indicators during CPET. After verifying the effectiveness of the designed model, the significance of the data from different phases in CPET for predicting the efficacy of AEI on BP lowering was further evaluated.

### 5.1. Description of the Dataset

(1) Inclusion criteria: between the ages of 18 and 45; stage I hypertension (SBP: 140–160 mmHg; DBP: 90–100 mmHg) either without medication or with discontinuation of antihypertensive drugs for more than two weeks and still presenting stage I hypertension; no regular exercise for four months prior to admission; willingness to participate in follow-ups for more than 6 months.
(2) Treatment prescription: patients underwent aerobic exercise with an Italian COSMED K4 electric bicycle. Training intensity corresponded to the metabolic equivalent of task (MET) of 70% of maximal oxygen consumption (VO_2max_). Get aerobic exercise 5 times per week, each time 45 minutes (exercise intensity equivalent to 2,000–3,000 kcal per week), lasting 12 weeks.
(3) Classification standard: patients were categorized as strong or weak responders of AEI treatment according to the therapeutic effect. The classification process is as follows:
  1. All patients received 24-hour dynamic BP monitoring before and after AEI to obtain their daily mean BP.
  2. The rate of BP change before and after treatment was calculated for each patient: *r*_*i*_=‖MBPB − MBPA‖/MBPB, where MBPB and MBPA indicated the mean BP of 24 hours before and after treatment, respectively.
  3. *Z*-score standardization was performed for *r*_*i*_ as follows: *z*_*i*_=(*r*_*i*_ − *μ*)/*σ*, where *μ* and *σ* were the mean and standard deviation, respectively. The role of *z*_*i*_ was to determine whether the antihypertensive efficacy of the *i*th patient was above average.
  4. Classify according to *z*_*i*_. Patients with *z*_*i*_ >0 (14 individuals in total) were identified as the strong antihypertensive responders of AEI, while patients with *z*_*i*_ <0 (10 individuals in total) were classified as weak responders. The real labels of 24 patients are detailed in Table 1.

As can be seen from Table 1, all patients except the last one exhibited certain antihypertensive effects following 12 weeks of AEI treatment. The average antihypertensive change rate was 7.582%. The individual showing the best antihypertensive effect exhibited a 40 mmHg (or 16.529%) BP decrease after AEI. However, the absence of obvious changes in BP of some individuals also proved that the efficacy of AEI is significantly different in hypertensive patients.

### 5.2. Experimental Results

In this paper, accuracy and F1-score (the harmonic average of precision and recall) obtained by the confusion matrix (see Figure 5) were used to evaluate the performance of the model. For them, higher values indicate positive benefits.

#### 5.2.1. The Performance of the Baseline Method Based on BP Change

An intuitive way to predict the BP-lowering effect of AEI is to determine whether the BP of patients after exercise is lower than that before exercising in CPET. Specifically, the pre-exercise resting BP (PEBP) was subtracted from BP at the 6th minute of the recovery phase (R6BP) to obtain BP change (△BP) for each patient. A patient with △BP less than 0 was considered to be unable to benefit from AEI, meaning the predicted label was weak. Conversely, a patient would exhibit a strong, beneficial antihypertensive response to AEI. The predicted labels of the baseline method based on BP change are shown in Table 2. Using the confusion matrix, the accuracy of the baseline method was 0.542, and F1-score was 0.56. This meant that the baseline method was only slightly superior to the random guess (accuracy = 0.5), far less than the requirement for clinical applications.

#### 5.2.2. The Performance of Machine Learning Models Based on the Metabolic Indicators

Time series of the nine metabolic indicators described above during the exercise phase were selected for analysis using machine learning models. Of note, patients had distinct exercise durations based on different physical conditions, resulting in different numbers of sampling points for individuals (ranging from 85 to 270). As most machine learning models required samples to have the same dimension, linear interpolation was first applied to unify the sampling numbers of all patients to 270 points. Afterward, SRC-AL presented herein was compared with SRC and some popular models of TSC, including 1NN-DTW, random forest (RF), and support vector machine (SVM). Due to the limited samples, the leave-one-out cross-validation was adopted to carry out the experiments [52]. All the above models were implemented by MATLAB. For SRC and SRC-AL, OMP and K-SVD algorithms in the SPAMS toolbox were used to solve the sparse representation and dictionary learning, respectively. Besides, the optimal sparse factor was obtained by grid search in a specific interval. Finally, for SRC-AL, the size of the initial dictionary was defined as a matrix where the number of columns was twice the number of rows, which was realized by the discrete cosine transform. The experimental results of each model are shown in Tables 3 and 4, where the last column of each table shows the average performance of each metabolic indicator based on different machine learning models.

#### 5.2.3. The Performance of SRC-AL Based on the Data from Different Phases of CPET

Since SRC-AL performed best in the above model, it was directly used to evaluate the significance of the data generated in the three important phases of CPET for predicting the individual responsiveness to AEI. These three phases included warm-up, exercise, and recovery. Similar to the exercise phase, the data dimensions of different patients in the other two phases were also inconsistent. For the warm-up phase, the shortest time series of metabolic indicators had only 38 sample values, while the longest had 81 sample values. For the recovery phase, the shortest one had only 113 sample values, while the longest one had 195 sample values. Therefore, linear interpolation should be used first to unify the data dimensions of different patients into the same. Besides, the dictionary learned in the exercise phase cannot be applied to the other two phases due to different data dimensions. The experimental results of SRC-AL based on the data of the above three phases of CPET are shown in Table 5.

### 5.3. Analyses of Experimental Results

This work investigated the ability of metabolic indicators to discriminate between strong and weak responses to AEI in patients. Through the analysis of the above experimental results, the following insights can be obtained to help clinicians predict the efficacy of AEI on young hypertensive patients based on CPET.

1. From Tables 3 and 4, SRC-AL and SRC were superior to other traditional classifiers in predicting the individual responsiveness to AEI based on the time series of metabolic indicators. This is mainly because the process of collecting these metabolic indicator data is prone to generate many interference signals, while the sparse representation can effectively extract the main features of time series and enhance the robustness to noise to the maximum extent.
2. The performance of SRC-AL was significantly better than that of SRC regardless of the time series based on any indicator, although both were based on sparse representation. This indicates that SRC needs an adequate set of training samples to form an overcomplete dictionary for better performance. On the contrary, SRC-AL can always guarantee the overcompleteness because it generates dictionaries employing the analytic approach. Through dictionary learning, the initial dictionary can be gradually updated to better fit the training samples and their labels.
3. According to the last column of Table 3, except for the indicator VE/VCO_2_, the average accuracy of all the other metabolic indicators based on the five machine learning models was higher than that of the baseline method based on BP change (accuracy = 0.542). However, if evaluated by the average F1-score, all metabolic indicators were superior to BP change alone (F1-score = 0.56), as shown in the last column of Table 4. This interesting finding suggests that the multipoint characteristics of cardiopulmonary metabolic indicators formed by collecting breath data can more accurately reflect the individual responsiveness to AEI.  Figure 6 visualizes the comparison between the predictive performance of each indicator obtained by machine learning models and that of BP change obtained by the baseline method, where Figure 6(a) shows the average/optimal accuracy and Figure 6(b) shows the average/optimal F1-score. Note that the optimal performance of all metabolic indicators was obtained by SRC-AL designed herein.
4. Table 5 illustrates the significance of data from different phases in CPET for predicting the BP-lowering effect of AEI. VO_2_/HR, VE, VO_2_/kg, VT, and R had the best predictive effect by using the time series of the exercise phase, while HR, SV, and VE/VCO_2_ performed better according to the time series of the warm-up phase. The performance of CO was consistent in both the exercise and the warm-up phases. Finally, the data in the recovery phase were less important than in the previous two phases. The reason may be that the patient is only active for the first three minutes during the recovery phase and remains inactive for the next three minutes. In other words, the metabolic data of patients in the active state are more significant for predicting the individual responsiveness to AEI.

### 5.4. Additional Experiments

Considering that the sample size of the aforementioned experiments is rather limited, six datasets from the UCR Time Series Classification Archive were selected for additional experiments to further verify the effectiveness of our proposed model [53]. The common characteristics of these datasets include the following: (1) the number of classes is two and (2) the number of training samples is less than or close to the length of the sample. This results in the dictionary based on data implementation not being overcomplete, which may reduce the classification accuracy of SRC. Nevertheless, the proposed model based on analytic dictionary learning (SRC-AL) should not be affected. The detailed description of the datasets is shown in Table 6. According to the results demonstrated in Table 7, SRC-AL achieved the best classification in all the datasets, indicating that SRC-AL is particularly suitable for datasets with fewer training samples than the sample length.

In addition, considering that SRC-AL is an extended sparse representation classifier, an interesting question is whether or not other machine learning models can be modified to handle the problem addressed in this paper with better performance. To answer this question, the improved versions of some machine learning models were used to be compared with SRC-AL. For example, in order to reduce the huge feature space of the random forest, time series forest (TSF) was used to divide a time series into $\sqrt{m}$ random intervals (*m* is the length of the time series), and then the mean, standard deviation, and slope of each interval were all taken as features for classification [54]. Similarly, in order to improve the classification accuracy of 1NN-DTW, 1NN-sharpDTW was first adopted to convert the time series into a sequence of shape descriptors, and then the locally similar structures were paired [55]. Aiming to extract different characteristics of the domain data, three description functions were utilized to encode local shape information in this paper: raw subsequence (RAWS), discrete wavelet transform (DWT), and slope. Specifically, RAWS was applied to directly take a subsequence of the data around a sampling point of a time series as its shape descriptor. On this basis, DWT was used to decompose each subsequence into three levels, and then all the coefficients were serialized into a shape descriptor. Alternatively, the slope function was first adopted to divide each subsequence into several intervals, and then the slopes of the fitting lines of all the intervals were concatenated into a shape descriptor. According to the results shown in Table 8, SRC-AL performed best in all the improved versions. This fully demonstrates the significance of sparse representation in feature extraction and noise reduction of CPET data.

## 6. Conclusions and Future Works

In recent years, the incidence of hypertension has shown a clear trend towards presenting in younger patients. Note that AEI has been recognized as an effective treatment among young hypertensive patients. Unfortunately, research regarding how to predict the individual responsiveness to AEI for young hypertensive patients is still lacking. As such, a sparse representation classifier based on analytic dictionary learning, a.k.a. SRC-AL, was designed to mine the time series of multiple cardiopulmonary metabolic indicators from CPET data to accurately estimate the effectiveness of AEI on patients' BP management.

In summary, the experimental results first showed that the machine learning model, especially SRC-AL, which is based on the time series of metabolic indicators, can better predict the individual responsiveness to AEI than the baseline method that is based on scalar values of BP change alone. Secondly, data from the exercise phase in CPET are the first choice for data mining, with the second choice being data from the warm-up phase. Thirdly, VO_2_/HR is strongly recommended as a powerful, new prognostic indicator for predicting aerobic exercise efficacy as an antihypertensive, with an average accuracy of about 75% and up to 100%. Besides, CO is also a good choice not only because its average performance is second only to VO_2_/HR but also due to the fact that its performance is very stable in both warm-up and exercise phases. As such, this will likely prove to be useful to clinicians for more accurately selecting comprehensive antihypertensive treatment measures without requiring extra clinical testing.

Note that the predictive model in this study is a qualitative prediction that predicts whether or not an individual hypertensive patient's response to aerobic exercise intervention is ideal. In future work, the quantitative prediction model of BP reduction caused by AEI is planned to be studied. Besides, BP defined in the current model is the sum of SBP and DBP. It may make more sense to analyze SBP and DBP separately in the subsequent work. Finally, the work presented here includes data generated from 24 young patients with stage I hypertension. Due to the limited sample size of this dataset, more samples should be collected in the future to prove the robustness of the proposed method. At the same time, further optimization can be attempted through the data augmentation technologies.

## Figures and Tables

**Figure 1:** Illustration of cardiopulmonary exercise testing. To protect privacy, the patient's eyes were partially blurred.

**Figure 2:** Visualization of several indicators for a patient during the exercise phase of a CPET. (a) Heart rate. (b) Stroke volume. (c) Cardiac output. (d) Oxygen pulse. (e) Oxygen consumption/kilogram. (f) Tidal volume. (g) Ventilation volume/minute. (h) Respiratory exchange ratio. (i) Carbon dioxide ventilation equivalent.

**Figure 3:** The SRC schematic for a two-class problem, where *y* is the unlabeled sample. *D*_1_ and *D*_2_ represent subdictionaries composed of all normalized samples belonging to class 1 and class 2, respectively. The sparse representation *α* can be divided into two subvectors (*α*_1_ and *α*_2_) according to the number of columns in *D*_1_ and *D*_2_. The black-filled blocks in *α* represent nonzero elements.

**Figure 4:** The SRC-AL schematic for a two-class problem, where *x*_1_ and *x*_2_ represent the samples of class 1 and class 2, respectively, and *y* is the unlabeled sample. Due to the limited space, only two labeled samples are drawn in the figure. In fact, all labeled samples are used for dictionary learning. *D*_*up*_' and *D*_*lw*_' represent the upper and lower parts of the learned dictionary. *α*_*x*1_, *α*_*x*2_, and *α*_*y*_ are the sparse representations of *x*_1_, *x*_2_, and *y* where the black-filled blocks represent nonzero elements.

**Figure 5:** Illustration of the confusion matrix.

**Figure 6:** Comparison between the predictive performance of each indicator obtained by machine learning models and that of BP change obtained by the baseline method. (a, b) The average and optimal performance of metabolic indicators, respectively.

**Table 1:** Real labels of 24 young patients with stage I hypertension.

Sample	MBPB (mmHg)	MBPA (mmHg)	*r*_*i*_ (%)	*z*_*i*_	Label
1	242	202	16.529	2.209	Strong
2	229	195	14.847	1.792	Strong
3	221	192	13.122	1.365	Strong
4	241	212	12.033	1.094	Strong
5	235	213	9.362	0.432	Strong
6	253	230	9.091	0.365	Strong
7	223	203	8.969	0.334	Strong
8	249	227	8.835	0.301	Strong
9	209	191	8.612	0.246	Strong
10	244	223	8.607	0.245	Strong
11	214	196	8.411	0.196	Strong
12	246	226	8.130	0.127	Strong
13	204	188	7.843	0.055	Strong
14	244	225	7.787	0.041	Strong
15	244	226	7.377	−0.060	Weak
16	231	214	7.359	−0.065	Weak
17	240	223	7.083	−0.133	Weak
18	231	215	6.926	−0.172	Weak
19	214	207	3.271	−1.079	Weak
20	221	214	3.167	−1.104	Weak
21	222	216	2.703	−1.220	Weak
22	211	208	1.422	−1.537	Weak
23	207	205	0.966	−1.650	Weak
24	207	208	0.483	−1.770	Weak

**Table 2:** Predicted labels of the baseline method based on BP change, where △BP = PEBP − R6BP.

Sample	PEBP (mmHg)	R6BP (mmHg)	△BP (mmHg)	Predicted label	Real label
1	242	267	−25	Weak	Strong
2	233	260	−27	Weak	Strong
3	199	170	29	Strong	Strong
4	236	216	20	Strong	Strong
5	190	223	−33	Weak	Strong
6	238	246	−8	Weak	Strong
7	209	205	4	Strong	Strong
8	274	256	18	Strong	Strong
9	201	203	−2	Weak	Strong
10	224	214	10	Strong	Strong
11	204	211	−7	Weak	Strong
12	262	255	7	Strong	Strong
13	216	218	−2	Weak	Strong
14	219	194	25	Strong	Strong
15	222	232	−10	Weak	Weak
16	245	229	16	Strong	Weak
17	247	250	−3	Weak	Weak
18	176	173	3	Strong	Weak
19	233	225	8	Strong	Weak
20	219	227	−8	Weak	Weak
21	205	206	−1	Weak	Weak
22	223	235	−12	Weak	Weak
23	216	242	−26	Weak	Weak
24	224	185	39	Strong	Weak

**Table 3:** Accuracy of various machine learning models based on the data from the exercise phase of CPET.

Indicator	SRC-AL	SRC	1NN-DTW	RF	SVM	Mean
VO_2_/HR	1.000	0.792	0.625	0.583	0.667	0.733
VE	0.875	0.708	0.625	0.458	0.542	0.642
VO_2_/kg	0.917	0.667	0.500	0.500	0.583	0.633
CO	0.917	0.667	0.500	0.583	0.792	0.692
HR	0.833	0.625	0.500	0.500	0.417	0.575
SV	0.667	0.542	0.458	0.542	0.542	0.550
VE/VCO_2_	0.708	0.542	0.500	0.458	0.458	0.533
VT	1.000	0.458	0.583	0.500	0.333	0.575
R	0.958	0.417	0.375	0.500	0.583	0.567

**Table 4:** F1-score of various machine learning models based on the data from the exercise phase of CPET.

Indicator	SRC-AL	SRC	1NN-DTW	RF	SVM	Mean
VO_2_/HR	1.000	0.815	0.667	0.667	0.714	0.773
VE	0.903	0.741	0.640	0.581	0.593	0.692
VO_2_/kg	0.933	0.692	0.539	0.600	0.643	0.681
CO	0.923	0.692	0.571	0.667	0.828	0.736
HR	0.846	0.640	0.539	0.600	0.462	0.617
SV	0.667	0.667	0.552	0.645	0.621	0.630
VE/VCO_2_	0.778	0.667	0.600	0.606	0.581	0.646
VT	1.000	0.381	0.615	0.571	0.429	0.599
R	0.966	0.462	0.516	0.571	0.643	0.632

**Table 5:** The performance of SRC-AL based on the data from the three phases of CPET.

Indicator	Warm-up accuracy	Exercise accuracy	Recovery accuracy	Warm-up F1-score	Exercise F1-score	Recovery F1-score
VO_2_/HR	0.583	1.000	0.625	0.737	1.000	0.743
VE	0.625	0.875	0.833	0.757	0.903	0.875
VO_2_/kg	0.750	0.917	0.750	0.824	0.933	0.824
CO	0.917	0.917	0.708	0.923	0.923	0.720
HR	0.833	0.833	0.792	0.857	0.846	0.828
SV	0.958	0.667	0.625	0.963	0.667	0.757
VE/VCO_2_	0.750	0.708	0.708	0.800	0.778	0.788
VT	0.583	1.000	0.792	0.737	1.000	0.828
R	0.917	0.958	0.708	0.923	0.966	0.759

**Table 6:** Brief description of six datasets from the UCR Time Series Classification Archive.

Type	Dataset	Classes	Length	Training set	Testing set
ECG	ECGFiveDays	2	136	23	861
ECG	ECG2000	2	96	100	100
Sensor	SonyAIBORobotSurface1	2	70	20	601
Spectro	Ham	2	431	109	105
Image	Herring	2	512	64	64
Image	BeetleFly	2	512	20	20

**Table 7:** Classification accuracy of various machine learning models on UCR datasets.

Dataset	SRC-AL	SRC	1NN-DTW	RF	SVM
ECGFiveDays	0.974	0.971	0.768	0.787	0.974
ECG2000	0.920	0.900	0.770	0.819	0.770
SonyAIBORobotSurface1	0.890	0.757	0.725	0.733	0.677
Ham	0.762	0.619	0.467	0.722	0.619
Herring	0.672	0.609	0.531	0.572	0.625
BeetleFly	0.900	0.650	0.700	0.825	0.900

**Table 8:** Accuracy of improved versions of various machine learning models based on the data from the exercise phase of CPET.

Indicator	SRC-AL	1NN-sharpDTW (RAWS)	1NN-sharpDTW (DWT)	1NN-sharpDTW (slope)	TSF
VO_2_/HR	1.000	0.625	0.583	0.542	0.675
VE	0.875	0.583	0.583	0.667	0.392
VO_2_/kg	0.917	0.458	0.500	0.500	0.450
CO	0.917	0.833	0.833	0.667	0.558
HR	0.833	0.500	0.542	0.542	0.517
SV	0.667	0.583	0.625	0.542	0.592
VE/VCO_2_	0.708	0.625	0.583	0.542	0.542
VT	1.000	0.542	0.542	0.625	0.392
R	0.958	0.583	0.583	0.625	0.517

## Data Availability

The data used to support the findings of this study cannot be made freely available in order to protect patient privacy. Requests for access to these data should be made to the corresponding author.
